# The Effect of Acupuncture Combined with Aerobic Exercise for Coronary Heart Disease as Cardiac Rehabilitation

This article has been retracted.

**DOI:** 10.1155/2022/4903265

**Published:** 2022-03-15

**Authors:** Yan Yang, Yaoyao Li, Yuanyuan Zheng, Lei Zhang, Wei Ma, Lingling Shi, Jingjing Kong, Xiaoli Liu, Hong Yu

**Affiliations:** Department of Cardiology, Shanghai Punan Hospital of Pudong New District, Shanghai 200125, China

## Abstract

**Background:**

The mortality of coronary heart disease continues to rise. Cardiac rehabilitation intervenes the risk factors of cardiovascular disease, improves cardiopulmonary function, maintains healthy psychology, improves the quality of life of patients, and reduces cardiovascular mortality.

**Objective:**

To explore the effect of acupuncture combined with aerobic exercise on cardiopulmonary exercise ability, blood lipid, fatty acid oxidation, and psychology in patients with coronary heart disease.

**Methods:**

Sixty patients with coronary heart disease from February 2018 to October 2020 were randomly divided into two groups: the control group and experimental group. The control group was given an exercise prescription, and the experimental group was given acupuncture combined with an exercise prescription. Before and after the intervention, the cardiopulmonary exercise test, blood lipid, carnitine acyltransferase (CACT), the Self-Rating Somatic Symptom Scale (SSS), the Generalized Anxiety Disorder-7 (GAD-7), and the Patient Health Questionnaire-9 (PHQ-9) of the two groups were compared.

**Results:**

The PHQ-9 score was better in the experimental group than in the control group. In both groups, after the intervention, the peak oxygen uptake and anaerobic threshold were increased, and blood lipid and PHQ-9 scores were decreased. In the experimental group, the carbon dioxide metabolic equivalent was decreased, CACT was increased, and SSS and GAD-7 scores were decreased, with statistical difference (*P* < 0.05).

**Conclusion:**

Acupuncture combined with aerobic exercise can improve the cardiopulmonary exercise ability, increase fatty acid oxidation, decrease blood lipid, and ameliorate anxiety and depression symptoms of patients with coronary heart disease as cardiac rehabilitation.

## 1. Introduction

Cardiovascular disease is the leading cause of disability and death in Chinese residents [1]. There are more than 11 million people suffering from Coronary Artery Atherosclerotic Heart Disease (CHD) in China [2]. Despite the continuous development of drugs and interventional therapy, the mortality of coronary heart disease in China continues to rise [3]. The substantial decline in mortality of coronary heart disease in developed countries is due to coronary heart disease rehabilitation and secondary prevention [4]. China urgently needs to strengthen the prevention and rehabilitation of cardiovascular diseases. Cardiac rehabilitation applied drugs, exercise, nutrition, and psychological and behavioural intervention to comprehensively intervene the risk factors of cardiovascular disease, improve cardiopulmonary function, maintain healthy psychology, improve the quality of life of patients, and reduce cardiovascular mortality [5–7].

Acupuncture, having bidirectional regulatory ability and a much lower incidence of side effects, can treat a variety of diseases. It can intervene hypertension and psychological stress-induced cardiovascular reactivity to prevent cardiovascular disease and cardiovascular death [8]. It has been used as adjuvant therapy for chronic stable angina pectoris, which can reduce the frequency of angina attacks [9]. This study observed the effect of acupuncture treatment on cardiopulmonary exercise ability, blood lipid metabolism, and psychology of patients with coronary heart disease and explored rehabilitation strategy suitable for China's national conditions.

## 2. Subjects and Methods

### 2.1. Subjects

This study included sixty patients with stable coronary heart disease who were admitted to the Department of Cardiology, Punan Hospital, Pudong New District, Shanghai, from February 2018 to October 2020. Inclusion criteria: age >18 years and <85 years, stability of symptoms and dose for at least 2 weeks; coronary angiography showed at least one major coronary artery stenosis >50%; and obtained consent and sign informed consent. Exclusion criteria: those who are unwilling or unable to exercise or acupuncture treatment; there has been acupuncture treatment in the recent 6 months; bone and joint diseases affecting movement; aortic dissection; acute coronary syndrome; uncontrolled heart failure; and severe liver and renal dysfunction. Using random numbers, 60 cases were divided into the control group and experimental group.

### 2.2. Methods

#### 2.2.1. Intervention Methods

All patients were treated with cardiac rehabilitation under the guidance of cardiac rehabilitation doctors. Exercise prescriptions were issued according to cardiopulmonary exercise test (CPXT). The control group received exercise rehabilitation, and the experimental group received acupuncture treatment and exercise rehabilitation. Exercise prescription: exercise intensity set anaerobic threshold heart rate as target heart rate; exercise frequency for 3–5 times a week, 20–30 minutes aerobic exercise, a total of 8 weeks; the form of exercise is mainly jogging and power cycling. Acupuncture acupoints were selected by acupuncture doctors according to the clinical symptoms of patients, and the selected acupoints were the following acupoint combinations. Chest discomfort acupoints: Nei guan, Ju Que, Shen men, Guan Yuan, Qi hai, and Da ling; insomnia acupoints: Bai hui, Zhao hai, and Tai Chong; shoulder pain acupoint: Jian yu, Jian Liao, Jian Zhen, Qu chi, and Wai guan; lower limb pain acupoint: Yin ling Quan, Chen shan, Tiao Kou, Zu san li, San yin jiao, Fu Tu, and Feng shi; and knee Joint pain acupoints: Nei Wai Xi Yan, Xue Hai, He Ding, Yang Ling Quan, etc. Acupuncture treatment was performed for 30 minutes each time, 1-2 times a week, for a total of 12 times.

#### 2.2.2. Cardiopulmonary Exercise Test (CPXT)

The Italian COSMED Cardiopulmonary exercise test system, exercise equipment for power cycling, with an increasing power (10–20 Watt Ramp) scheme for the symptom-limited maximum exercise load test, the V-slop method was used to calculate the anaerobic threshold (see Table 1).

#### 2.2.3. Biochemical Indicators

All patients were taken fasting venous blood, Abbott C16000 automatic biochemical analyzer for blood lipid testing, triglycerides with the GPO-PAP method, total cholesterol with the enzyme method, low-density lipoprotein with the direct method-surfactant clearance method, high-density lipoprotein with the direct method-selective inhibition method, free fatty acids with the ACS-ACOD method, blood glucose with the glucose oxidase method, serum creatinine with the enzyme method, the uric acid kinase method, and homocysteine with the double-reagent circulation enzyme method. Glycosylated haemoglobin was measured by using the Arkray 8180 instrument and high-performance liquid chromatography. Serum CACT was determined by using the ELISA kit. The kit was provided by Shanghai Kamishu Biotechnology Co., Ltd.

### 2.3. Observation Indicators

#### 2.3.1. CPXT Indicators

The CPXT indicators were peak oxygen uptake per kg body weight (VO2/kg), anaerobic threshold (AT) oxygen uptake, respiratory reserve, oxygen pulse, one-minute heart rate recovery, anaerobic threshold carbon dioxide ventilation equivalent (VE/VCO2 @ AT), and others.

#### 2.3.2. Biochemical Indicators

The biochemical indicators were serum creatinine, uric acid, triglyceride, cholesterol, low-density lipoprotein, high-density lipoprotein, free fatty acids, serum carnitine acyltransferase, blood glucose, glycosylated haemoglobin, blood homocysteine, etc.

#### 2.3.3. Psychological Assessment

Before and after the intervention, patients were asked to fill out the Self-Rating Somatic Symptom Scale (SSS), PHQ-9 health questionnaire (depression screening scale), and GAD-7 generalized anxiety disorder scale for psychological assessment.

### 2.4. Statistical Method

SPSS22.0 software was used. The measurement data were expressed as mean ± standard deviation, which was in line with normal distribution. A paired *t*-test was used for intragroup comparison, and an independent-sample *t*-test was used for intergroup comparison. Enumeration data were expressed as frequency and percentage. The Chi-square test was used for comparison between groups. *P* < 0.05 indicated statistical difference.

## 3. Results

### 3.1. Comparison of Baseline Basic Data between the Two Groups of Patients

There was no significant difference in gender, age, body mass index, history of hypertension, history of diabetes, homocysteine, creatinine, uric acid, triglyceride, cholesterol, low-density lipoprotein, high-density lipoprotein, free fatty acid, blood glucose, glycosylated haemoglobin (HbA1c), and other biochemical indicators between the two groups (*P* > 0.05), as shown in Table 2.

### 3.2. Comparison of the Cardiopulmonary Exercise Test

There was no significant difference between the two groups before and after intervention (*P* > 0.05). The peak oxygen uptake per kilogram (VO2/kg peak) and anaerobic threshold (VO2/kg @ AT) in the two groups were increased after intervention. The carbon dioxide ventilation equivalent (VE/VCO2 @ AT) in the experimental group decreased after intervention, with statistical significance (*P* < 0.05).

### 3.3. Comparison of Biochemical Indicators

There was no significant difference between the two groups in serum creatinine, uric acid, triglyceride, high-density lipoprotein, free fatty acid, blood glucose, glycosylated haemoglobin, and other biochemical indicators before and after intervention (*P* > 0.05). Compared within the group, the low-density lipoprotein and cholesterol in the two groups decreased after the intervention, and the serum carnitine acyltransferase in the experimental group increased after intervention, with a statistical difference (*P* < 0.05) (Table 3).

### 3.4. Comparison of Psychological Scales between the Two Groups

There was no significant difference between the two groups before intervention. After intervention, the acupuncture group improved PHQ-9 compared with the control group (*P* < 0.05). Compared within the group before and after intervention, the acupuncture group improved the Chinese somatization symptom checklist, PHQ-9 and CAD-7, and aerobic exercise improved PHQ-9 (*P* < 0.05), see Table 4.

## 4. Discussion

This study shows that aerobic exercise can improve peak oxygen uptake and anaerobic threshold in patients with coronary heart disease and reduce blood lipids. Aerobic exercise increases ventricular end-diastolic volume, myocardial contractility, and cardiac output through the sympathetic nerve and improves coronary artery circulation by increasing nitric oxide production and vasodilation; exercise can also reduce blood lipids and inflammation indicators [10]. Therefore, exercise is good medicine for heart rehabilitation. Based on a large number of clinical studies and systematic evaluation results in China, Europe, the United States, and other countries, guidelines for the prevention and rehabilitation of cardiovascular diseases based on exercise are introduced [11, 12].

This study found that acupuncture in the rehabilitation of patients with coronary heart disease can also bring three other benefits.

Fatty acid is an important source of muscle contraction energy, acetyl-CoA fatty acid is tranfered by the carnitine palmitoyl transferase system into mitochondrial oxidation. This study suggests that acupuncture can increase the concentration of serum carnitine acyltransferase, infer acupuncture promote fatty acid oxidation, and enhance myocardial and skeletal muscle energy supplement. Glucose is the main energy source during embryogenesis, and fatty acid oxidation is the main energy source after birth. The selection and change of myocardial energy substrates are the objects of myocardial metabolise in patients with ischemic heart disease and heart failure. Energy utilization efficiency and myocardial efficiency is a potential target for the treatment of heart failure and ischemia [13]. Animal experiments have found that the lack of carnitine palmitoyltransferase can lead to cardiac hypertrophy due to excessive pressure load caused by lipotoxicity [14]. Acupuncture treatment can regulate heart energy metabolism by affecting the key enzymes of fatty acid metabolism, with fewer adverse reactions and high safety.

Carbon dioxide ventilation equivalent (VE/VCO2) is the most widely studied ventilation efficiency parameter. The increase in VE/VCO2 is significantly associated with the mortality of patients, which is a reliable indicator for the prognosis of heart failure [15]. In this study, it was found that acupuncture treatment could reduce the anaerobic threshold carbon dioxide ventilation equivalent (VE/VCO2 @ AT), which was similar to the previous research results of acupuncture treatment for patients with heart failure in Germany [16]. The increase of VE/VCO2 was due to the increase of invalid ventilation residual cavity, mismatch of blood flow and ventilation, a decrease of skeletal muscle oxidation ability, and an increase of exercise lactic acid to stimulate breathing. Previous studies have found that acupuncture can reduce the production of lactic acid during exercise [17]. This study found that acupuncture can enhance fatty acid oxidation, so it is speculated that these two factors are the reasons why acupuncture can reduce VE/VCO2. Lowering VE/VCO2 may benefit, especially, cardiovascular patients who cannot exercise and have a poor response to treatment, suggesting that acupuncture can be used as a choice for rehabilitation.

Psychological anxiety, depression, and other emotional factors are not only risk factors for coronary heart disease but also closely related to the development of coronary heart disease. A systematic review [18] shows that exercise therapy may reduce depressive symptoms, while anxiety symptoms may be reduced in the short term (less than 12 weeks) and long-term outcomes are uncertain. By literature analysis [19] from 2011 to 2020, more and more studies have shown that acupuncture can be used as a potentially effective treatment for depression and improve depressive symptoms. Acupuncture treatment has positive results in the treatment of anxiety [20]. Metabonomics technology is used to analyze the body metabolism by acupuncture and moxibustion, which shows that acupuncture and moxibustion canchange plasma tryptophan and glutamate, regulate neurotransmitter, improve function, and promote health [21].

Acupuncture is based on the meridian theory, a guide for TCM dorctors to treat diseases, but the mechanism of acupunture is still unclarified; animal experiments have found that acupuncture activates the peripheral sensory nerve fibres of dorsal root ganglion and transmits the signals to the spinal cord and brain, thereby activating the peripheral autonomic nerve. Stimulating the acupoints of hind limbs (Zusanli) in mice can activate the vagal-adrenal anti-inflammatory pathway [22, 23]. Acupuncture and moxibustion activate the vagus nerve, reduce visceral immune cell production factors, reduce inflammatory factors, inhibit sympathetic nerve, and regulate neurohumoral factors, which can theoretically play more roles in cardiovascular diseases.

Therefore, acupuncture can improve the efficiency of exercise ventilation,promote fatty acid oxidation, improve anxiety and depression symptoms, and treat somatization symptoms in patients with coronary heart disease; combined with aerobic exercise can improve the cardiopulmonary exercise ability of patients and reduce blood lipids, which can be applied as cardiac rehabilitation technology.

The shortcomings of this study: (1) failure to set up a sham acupuncture control group because it was difficult to select acupoints in the sham acupuncture group during the preexperiment; (2) also, because there is no effect, patient compliance is not high in the sham acupuncture group after completing 1-2 times; and (3) the number of cases enrolled in this study is small; subsequent studies can expand the sample size and improve follow-up time to assess the long-term efficacy of acupuncture.

## Figures and Tables

**Table 1:** Comparison of cardiopulmonary exercise parameters between the two groups of patients with coronary heart disease after and before treatment (mean ± standard deviation).

Groups	Cases	VO_2_/kg peak （mL/min/kg）		VO_2_/kg@AT （mL/min/kg）		VE/VCO_2_@AT	
		Before treatment	After treatment	Before treatment	After treatment	Before treatment	After treatment
Trial groups	30	15.66 ± 4.63	16.75 ± 4.17 ^*∗*^	12.64 ± 3.75	15.07 ± 4.09 ^*∗*^	34.54 ± 5.98	32.89 ± 5.84 ^*∗*^
Control groups	30	15.82 ± 2.46	18.45 ± 3.53 ^*∗*^	12.91 ± 1.76	16.60 ± 3.88 ^*∗*^	33.23 ± 3.01	33.49 ± 2.66
*t* value		−0.122	−1.231	−0.265	−1.033	0.781	−0.355
*P* value		−0.904	0.228	0.794	0.311	0.443	0.726

Compared with before treatment,  ^*∗*^*P* < 0.05.

**Table 2:** Basic information of the two groups.

	Acupuncture groups	Control groups
Number of people	30	30
Male	20	16
Age (years)	58.94 ± 13.53	62.60 ± 17.54
BMI (kg/m^2^)	25.03 ± 3.39	24.83 ± 2.90
Hypertension	22	20
Diabetes	17	14
Homocysteine, umol/L	13.66 ± 11.39	11.39 ± 3.28
Creatinine, umol/L	70.71 ± 14.62	68.46 ± 17.51
Uric acid, umol/L	319.86 ± 62.71	313.46 ± 47.34
Triglyceride, mmol/L	1.53 ± 1.08	1.70 ± 0.54
Cholesterol, mmol/L	4.20 ± 1.32	4.70 ± 1.00
Low-density lipoprotein(LDL), mmol/L	2.69 ± 1.03	2.60 ± 0.79
High-density lipoprotein (HDL), mmol/L	1.08 ± 0.27	1.01 ± 0.24
Free fatty acid, umol/L	503.23 ± 195.96	598.31 ± 292.91
Blood glucose, mmol/L	6.5 ± 1.92	5.65 ± 0.90
HbA1c, %	6.99 ± 1.36	6.23 ± 1.17

**Table 3:** Comparison of blood cholesterol, low-density lipoprotein, and serum carnitine acyltransferase between the two groups (mean ± standard deviation).

Groups	Cases	Low-density lipoproteins		Cholesterol		Serum carnitine acyltransferase enzyme U/L	
		Before treatment	After treatment	Before treatment	After treatment	Before treatment	After treatment
Acupuncture group	30	2.69 ± 1.03	1.88 ± 0.67 ^*∗*^	4.20 ± 1.32	3.5 ± 1.04 ^*∗*^	189.09 ± 58.13	216.64 ± 57.36 ^*∗*^
Control group	30	2.60 ± 0.79	2.10 ± 0.54 ^*∗*^	4.70 ± 1.00	3.89 ± 0.58 ^*∗*^	202.45 ± 60.83	208.60 ± 56.48
*t* value		0.274	−2.092	−1.128	−1.074	−7.13	0.45
*P* value		0.786	0.059	0.27	0.293	0.48	0.65

**Table 4:** Comparison of the two groups' psychological self-rating scale (mean ± standard deviation).

Groups	Cases	Somatic self-rating scale		PHQ-9		CAD-7	
		Before treatment	After treatment	Before treatment	After treatment	Before treatment	After treatment
Acupuncture groups	30	34.5 ± 5.98	32.89 ± 5.84 ^*∗*^	4.91 ± 3.56	2.1 ± 1.85 ^*∗*^	4.72 ± 5.04	1.54 ± 1.84 ^*∗*^
Control groups	30	33.23 ± 3.01	33.49 ± 2.66	5.4 ± 3.06	4.3 ± 2.71 ^*∗*^	3.30 ± 4.19	2.8 ± 3.22
*t* value		0.781	−0.355	−0.337	−2.119	0.701	−1.107
*P* value		0.443	0.726	0.74	0.048	0.492	0.283

Compared with before treatment,  ^*∗*^*P* < 0.05.

## Data Availability

Data supporting the results of the study can be obtained by emailing the first author or corresponding author.
